# Prediction of Automobile Wiper Motor Noise Based on Support Vector Machine with Vibration Sensors

**DOI:** 10.1155/2022/3873651

**Published:** 2022-03-31

**Authors:** Haiqing Li, Zhanhao Cui, Yudong Wu, Xiaguang Ren, Ting Zhao

**Affiliations:** ^1^Liuzhou Vocational and Technical College, Liuzhou 545006, China; ^2^National Laboratory for Rail Transportation, Southwest Jiaotong University, Chengdu 610031, China

## Abstract

Wiper motor noise has an important impact on vehicle comfort. Accurate prediction of wiper motor noise can obtain motor NVH performance in motor manufacturing or earlier stage and provide necessary support for NVH performance design of parts and vehicles. However, the prediction accuracy of wiper motor noise by the traditional CAE or testing method is low. Data-driven technology provides a new idea for wiper motor noise prediction with its advantages of high efficiency and high precision. This paper studies the wiper motor noise prediction algorithm based on the motor vibration signal, respectively, using the transmission path analysis theory and the support vector machine theory, and carries on the test verification and comparative analysis of the effect. The results show that the method based on support vector machine is more accurate in the prediction of wiper motor noise and has higher practical engineering value.

## 1. Introduction

With the continuous upgrading of consumption in the automobile industry, consumers are paying more and more attention to the performance of noise, vibration, and harshness (NVH) of automobiles. Comprehensive performance parameter testing standards focus on increasingly stringent requirements for vibration and noise [1]. Automobile wiper is not only one of the key safety parts of the automobile but also has a huge impact on the comfort of the car. Accurately predicting the noise of the wiper motor can optimize the NVH performance of the motor in the manufacturing or earlier stages. Therefore, the accuracy and efficiency of automobile wiper motor noise prediction have high engineering practical significance for NVH performance design of components and vehicle system [2, 3].

The main components of motor noise of automobile wiper are electric drive system noise and structural sound radiation, and the electric drive system noise is composed of motor noise and transmission noise. The existing research on motor noise prediction mainly adopts CAE calculation method. Firstly, the motor structure model is established, and the modal frequencies and modal shapes of each order of the motor are calculated. After that, the electro-mechanical force is calculated through finite element analysis, and then the sound pressure level of motor noise is calculated with the help of commercial software such as ANSYS and LMS Virtual.Lab [4–9]. The mechanism of motor noise can be analyzed and optimized by CAE calculation method, but its prediction accuracy depends on the accuracy of various parameters of the motor, and the analysis process is heavy and the prediction cycle is long. The transfer path analysis method is applied to motor noise prediction, which dilutes the research on the mechanism of motor noise and directly establishes the connection between vibration and sound pressure, which can realize the rapid prediction of motor noise. In the background of the development of data-driven technology, the relationship between vibration and sound pressure is established through data mining, which provides a new idea for motor noise prediction [10, 11].

In this paper, the transmission path analysis method is used to study the noise transmission characteristics of automobile rear wiper motor and calculate the radiated noise. After obtaining a certain amount of data, a noise prediction model is established by data-driven method, and the connection among noise, vibration, and skeleton function is established by using support vector machine to predict motor noise.

## 2. Prediction Methods

### 2.1. Prediction Based on Traditional Transfer Path Analysis

TPA (transfer path analysis) is an analysis method based on source-path-receiver model, which is used to trace the root cause of vibration and noise [12, 13]. It has been widely used in the field of vehicle NVH and is an effective method to solve vehicle NVH problems. TPA methods are mainly divided into TPA in the time domain and TPA in the frequency domain. In both cases, the inverse matrix method is used to multiply the response of the indicating point by the inverse matrix of the frequency response function matrix to obtain the excitation force [14, 15]. The response of the target point can be expressed as follows:

(1) $$\begin{array}{c} P\left(\omega \right)=\sum_{i}{\text{NTF}}_{i}\left(\omega \right)F_{i}\left(\omega \right)+\sum_{j}{\text{NTF}}_{j}\left(\omega \right)Q_{j}\left(\omega \right), \end{array}$$

where *P*(*ω*) is the total sound pressure of the target point, *F*_*i*_ represents the structural load on the transmission path *i*, *Q*_*j*_ represents the acoustic load on the transmission path *j*, and NTF_*i*_ and NTF_*j*_ represent the transfer function of the corresponding path, respectively [12, 16].

In TPA analysis, the inverse matrix method (as shown in Figure 1) uses the transfer function VTF and the response signal of the passive part of the motor to inversely calculate the excitation force under the working state of the motor. At the same time, by measuring the transfer function NTF from the excitation point to the target point, the transfer relation between the motor excitation force and the sound pressure at the human ear is established, so as to realize the calculation of the noise at the human ear.

Operational path analysis (OPA) is a method used entirely in the operating state of a mechanical system [17, 18]. The analysis process only measures the operating condition data, without measuring the frequency response function at any position. The application of the transmissibility concept in OPA-based approaches is the major alternative to TPA, which provides a different solution by significantly reducing complexity and measurement time [19]. OPA analysis calculates the noise at the ear directly by estimating the transmissibility of the sound pressure signal transmitted from the motor vibration signal to the ear. Based on the calculation criterion of transmissibility, the response of the target point is expressed as the combined form of the response of the load position under the same working condition, so as to derive the analysis result similar to TPA. The response of the target point is shown in the following formula:

(2) $$\begin{array}{c} P\left(\omega \right)=\sum_{i}T_{i}\left(\omega \right){\ddot{X}}_{pi}\left(\omega \right)+\sum_{j}T_{j}\left(\omega \right)P_{j}\left(\omega \right), \end{array}$$

where *P*_*j*_ refers to the working sound pressure of the sound source, ${\ddot{X}}_{pi}\left(\omega \right)$ refers to the working acceleration response of the structure transfer path along the passive part, and *T*_*i*_ and *T*_*j*_ represent the transfer rates of sound pressure and acceleration between the target point and the loading position of the working load, respectively [20].

### 2.2. Prediction Based on SVM

Support vector regression algorithm is a machine learning method based on statistical learning theory and result risk minimization principle, which can solve small sample problems well [21, 22]. Support vector regression is divided into linear regression and nonlinear regression. In practical application, data are often not linearly separable. Support vector machine maps input *x*_*i*_ to a high-dimensional feature space through nonlinear mapping [23–25] and then constructs a linear model in this feature space. The mapping process is shown in Figure 2 and calculated by the following formula:

(3) $$\begin{array}{c} f\left(x\right)=\sum_{i=1}^{d}\omega_{i}\varphi_{i}\left(x\right)+b, \end{array}$$

where *d* is the dimension of the characteristic space, *φ*_*i*_(*x*) represents the nonlinear mapping, *ω*_*i*_ is the coefficient, and *b* is the deviation term. Different from the traditional regression model, support vector regression can tolerate the maximum *ε* deviation between the regression value *f*(*x*) and the actual value *y*. The loss is calculated when |*f*(*x*) − *y*| > *ε*, as shown in the following formula:

(4) $$\begin{array}{c} L_{\varepsilon }\left(y,f\left(x\right)\right)=\left\{\begin{array}{cc} 0, & \left|y-f\left(x\right)\right|\leq \varepsilon ,\\ \left|y-f\left(x\right)\right|-\varepsilon , & \text{otherwise,} \end{array}\right) \end{array}$$

where *L*_*ε*_ is the insensitive loss function, *ε* is the preset threshold value, and an interval band of width 2*ε* is constructed with *f*(*x*) as the center. If the sample falls into the interval band, its classification is correct. Using insensitive function in the feature space to linear regression, and by minimizing the ‖*ω*‖^2^ to reduce the complexity of the model, support vector regression method can be expressed as solving the following optimization problem, as shown in the following formula:

(5) $$\begin{array}{c} \underset{w,b}{\text{min}}\frac{1}{2}{\left\|\omega \right\|}^{2}+C\sum_{i=1}^{m}L_{\varepsilon }\left(y,f\left(x\right)\right), \end{array}$$

where *C* is the regularization parameter used to control the compromise between model complexity and approximation error, and *m* is the number of support vectors. The kernel function *K*(*x*_*t*_, *x*) is used to avoid the calculation of mapping function *φ*_*i*_(*x*) and reduce the computational complexity of high-dimensional hidden space.

## 3. Prediction Model Design and Wiper Motor Noise Test

### 3.1. Transfer Path Analysis Model

TPA analysis requires that the number of indicator points should be at least twice the number of paths. The establishment of TPA analysis model requires that on the basis of obtaining motor vibration and sound pressure signals, the transfer function VTF from motor excitation point to passive part and the transfer function NTF from human ear should be measured by hammer method. The excitation force of the motor on the excitation point is calculated to predict the noise at the ear. OPA analysis only needs to measure the working condition data, calculate the transmissibility through the vibration and sound pressure signals of the motor during operation, and establish the OPA analysis model. The noise prediction and analysis process of rear wiper motor based on transfer path analysis is shown in Figure 3.

### 3.2. Establishment of SVR Prediction Model

The collected test data were classified and all data were divided into training set and test set. In order to avoid using the same data as the test set in the training set, the test data of motor A was selected as the training set, and the test data of motor B was selected as the test set. Different motors have different excitation characteristics, and the problem frequency and peak value are changed, which ensures the uniqueness of test set data and the generalization ability of model.

In this paper, the Gaussian radial basis function is chosen as the kernel function of the SVR model. The penalty parameter *c* and the internal parameter *g* of the radial basis function are very important to the model, and the best *c* and *g* parameters are obtained by cross-validation and grid search in MATLAB. The input parameters of SVR model are variables of five dimensions, among which the three-way vibration acceleration signal of active point A occupies three dimensions, and the frequency point and the calculation results of sound pressure analyzed by OPA occupy one dimension, respectively. The output parameter of the model is a one-dimensional variable, that is, the sound pressure level near the ear. The inputs and outputs of the SVR model are shown in Figure 4.

SVR method uses data to drive noise prediction. From the perspective of acoustic vibration isolation, vibration data is the variable that can best establish connection with sound pressure data. Therefore, the three-way vibration acceleration of the active part measurement point is selected as the input parameter. We also used vibration signals of both active and passive part as input parameters to make noise prediction, but the prediction result was not improved compared with the model with only active part data, so the vibration data of passive part was not included in the SVR model. When training SVR models, one model training is adopted for every 1000 Hz frequency range, so frequency is taken as one of the input parameters. In addition, the OPA analysis results are put into the SVR model as one-dimensional input, because OPA analysis can be calculated using existing data without additional function transfer test, and the OPA method includes the mechanism of noise generation, which improves the accuracy of SVR model. However, after acquiring more test data, the SVR model can automatically mine the deep relationships between the data, without necessarily using OPA analysis results.

In order to prevent the values with large influence on the dependent variable from being masked, the input and output parameters are normalized in the range of [−1, 1], and the normalization equation is shown as follows:

(6) $$\begin{array}{c} x^{*}=2*\frac{x-x_{\min}}{x_{\max}-x_{\min}}-1, \end{array}$$

where *x*_max_ and *x*_min_ represent the maximum and minimum values in the data set, respectively; *x* and *x*^*∗*^ represent the values before and after normalization, respectively.

When training the SVR prediction model, it is important to balance the accuracy and efficiency of the model. Mean absolute error (MAE) was used to evaluate the accuracy of the prediction model, and the MAE calculation formula is shown in the following formula:

(7) $$\begin{array}{c} \text{MAE}=\frac{\sum_{i=1}^{n}\left|y_{i}-{\hat{y}}_{i}\right|}{n}, \end{array}$$

where *n* is the total number of frequency points, *y*_*i*_ is the test value of sound pressure level at the *i*th frequency point, and ${\hat{y}}_{i}$ is the predicted value of sound pressure level at the *i*th frequency point. If the prediction accuracy does not meet the requirements, the SVR model needs to be adjusted and the training samples need to be relearned. Model training flow chart is shown in Figure 5.

### 3.3. Wiper Motor Noise Test

The model used for the test was the LYNK and CO O2, and the test motor was a rear wiper motor. According to the needs of the transmission path analysis model, a three-way vibration acceleration sensor is arranged at the active part of the motor and two three-way vibration acceleration sensors are arranged at the passive part of the motor. The active part sensor is attached to the motor gearbox housing, and the passive part sensor is attached to the rear glass outside. The sound pressure sensor is arranged at the right ear of the driver. Sensors used in noise test are shown in Table 1. The sampling frequency is set to 12800 Hz and the sensor placement position is shown in Figure 6. TPA analysis requires testing the transfer function from the motor excitation point to the passive part and the human ear, where the NTF measured by the hammering method to the human ear is shown in Figure 7.

A motor and B motor were tested, respectively, and vibration and sound pressure data of the motor were collected under the condition of smooth operation. The sampling time was 3 s and the test times were 10 for each. After processing the test data and comparing the frequency spectrum of sound pressure values of motors A and B under the condition of smooth operation, it can be found that the problem frequency of noise generated by the two motors and the peak value at the problem frequency are significantly different. The comparison results are shown in Figure 8. On the premise that the noise characteristics of two motors are different, the TPA model and SVR model are established by using the test data of motor A to predict the noise characteristics of motor B.

## 4. Results and Discussion

The excitation force of motor B calculated by TPA analysis model during its smooth operation is shown in Figure 9, and the sound pressure level at the ear is predicted. The predicted results and the actual measurement results are shown in Figure 10(a). The transmissibility of motor during smooth operation is calculated from the test data of motor A, as shown in Figure 11. After the OPA analysis model is established, the sound pressure level near human ear during motor B is predicted. The predicted results and actual measurement results are shown in Figure 10(b). Based on the existing working data of motor A, the SVR model was trained and the noise of motor B was predicted. The comparison between the prediction results of SVR model and the actual measurement results is shown in Figure 10(c).

The accuracy of the prediction model was evaluated from two aspects of peak error and MAE, and the comparison results are shown in Table 2. The three models can predict the peak frequency well and find the problem frequency that affects the motor noise. The prediction error of OPA model at the peak frequency is obviously better than that of TPA model and SVR model. The mean square error of SVR model is smaller, and the overall trend is more consistent with the test results.

In the noise spectrum, frequencies with larger amplitude contribute more to noise and are often the key frequencies causing auditory discomfort, which is also the focus of NVH optimization. The rear wiper motor generates noise peak near 440 Hz, which is caused by vibration peak and transfer function peak alone or together. In terms of the prediction results at the peak, OPA method is obviously superior to TPA and SVR, which is related to the mechanism of the prediction method. TPA and OPA methods need to establish the transfer function from excitation to response to predict noise through noise generation mechanism, while TPA method limited by the transfer path in analysis may cause path omission, resulting in TPA prediction results lower than the actual value. The OPA method directly establishes the function of working condition without causing the omission of path. SVR method establishes the connection between vibration and noise through data-driven method, without solving the structural transfer function, which may result in low prediction results at the peak. However, with the increase of data volume, SVR model can mine the deep relationship between data and reflect the transfer mechanism in model parameters, and the prediction accuracy will gradually improve.

## 5. Conclusions

In this paper, the transmission path analysis method and support vector machine were used to establish the motor noise prediction model of the rear wiper motor, and the motor noise level was predicted. The accuracy of the prediction model was verified by experiments. Compared with the experimental results, it can be seen that these methods can accurately predict the problem frequency of motor noise. The prediction model based on OPA has a better prediction result at the peak, while the prediction model based on support vector machine has a higher overall prediction accuracy. Data-driven prediction models acquire knowledge from data. With the increase of the quantity and quality of test data, this method has greater development potential in prediction accuracy and efficiency.

## Figures and Tables

**Figure 1:** TPA inverse matrix.

**Figure 2:** Mapping to higher dimensions in SVM.

**Figure 3:** Transfer path analysis process.

**Figure 4:** The inputs and outputs of the SVR model.

**Figure 5:** SVR model training process.

**Figure 6:** Sensor position diagram.

**Figure 7:** Transfer function from excitation point to ear.

**Figure 8:** Comparison of noise characteristics between two motors.

**Figure 9:** Force excitation signal.

**Figure 10:** Working condition transmissibility.

**Figure 11:** Prediction results. (a) TPA method, (b) OPA method, and (c) SVR method.

**Table 1:** Sensors used in noise test.

Sensor type	Microphone	Accelerometer
Model	PCB 378B02	PCB 356A02
Sensitivity	50 mV/Pa	10 mV/g
Frequency range	3.75 to 20000 Hz	1 to 20000 Hz
Mass loading	45.8 g	10.5 g

**Table 2:** Noise prediction result comparison table.

Test and prediction method	Peak error (dB(A))	MAE (dB(A))
TPA	7	4.67
OPA	0.5	4.58
SVR	6	3.14

## Data Availability

The date used to support the findings of this study are available from the corresponding author upon request.
